# lncRNA ROR and miR-125b Predict the Prognosis in Heart Failure Combined Acute Renal Failure

**DOI:** 10.1155/2022/6853939

**Published:** 2022-01-20

**Authors:** Qianlong Xue, Lipeng Yang, Jia Wang, Linlin Li, Hui Wang, Ying He

**Affiliations:** ^1^Department of Emergency Medicine, The First Affiliated Hospital of Hebei North University, Zhangjiakou, China; ^2^Department of Gynecology, The First Affiliated Hospital of Hebei North University, Zhangjiakou, China

## Abstract

**Objective:**

To elucidate the correlation between expression levels of long noncoding RNA (lncRNA) ROR and microRNA-125b (miR-125b) with the prognosis in heart failure (HF) patients combined acute renal failure (ARF).

**Methods:**

HF patients combined ARF (*n* = 90) and healthy controls (*n* = 90) in the same period were included in our hospital from April 2016 to December 2018. Every subject was followed up for 24 months. Serum levels of lncRNA ROR and miR-125b were detected, and their expression correlation was analyzed by Pearson correlation test. Receiver operating characteristic (ROC) curves were depicted for assessing the sensitivity and specificity of lncRNA ROR and miR-125b in diagnosing HF combined ARF.

**Results:**

lncRNA ROR was upregulated in serum of HF patients combined ARF, and its level was positively correlated to NYHA classification. miR-125b displayed an opposite trend. In serum samples of HF combined ARF, expression level of lncRNA ROR was negatively related to that of miR-125b. Diagnostic potentials of lncRNA ROR and miR-125b in HF combined ARF were confirmed by ROC curve analyses (lncRNA ROR: AUC = 0.9199, cutoff value = 5.595, sensitivity = 92.22%, and specificity = 73.33%; miR-125b: AUC = 0.8509, cutoff value = 2.290, sensitivity = 81.11%, and specificity = 74.44%). After 2-year follow-up, 16 cases were dead. Higher incidences of death and rehospitalization were observed in HF combined ARF cases expressing higher serum level of lncRNA ROR or lower level of miR-125b.

**Conclusions:**

Serum level of lncRNA ROR is upregulated, and miR-125b is downregulated in HF patients combined ARF. Their levels are linked to NYHA classification, which can be utilized as prognostic biomarkers in HF combined ARF.

## 1. Introduction

Heart failure (HF) is caused by increased cardiac load and dyscirculatory syndrome owing to systolic and diastolic dysfunctions. As the heart disease worsens, insufficient blood perfusion and renal blood stasis impairs renal function [1]. Acute renal failure (ARF) is a clinical syndrome of rapid decline of glomerular filtration function, imbalance of water and electrolyte, and accumulation of nitrogen wastes in the body in a short period of time [2]. Clinically, HF patients are prone to develop ARF. ARF-induced water retention seriously continues to aggravate HF, thus increasing treatment difficulty [3].

Long noncoding RNAs (lncRNAs) are functional RNAs with over 200 nt long. They are generally transcribed in eukaryotes and unable to encode proteins [4]. Initially, lncRNAs were considered as byproducts of RNA polymerase II transcription without biological functions. Later, accumulating evidences have proven the vital functions in genomic imprinting, chromatin modification, transcriptional activation, and nuclear transportation at multiple levels [5]. In recent years, lncRNAs are reported as important regulators in HF [6]. Further, lncRNA ZNF593-AS alleviates contractile dysfunction in dilated cardiomyopathy [7]. And lncRNA H19 alleviates muscular dystrophy by stabilizing dystrophin [8]. lncRNA ROR locates on human chromosome 18q21.31 containing 4 exons [9]. Numerous previous studies have demonstrated the vital role of ROR in cardiovascular diseases. It is reported that lncRNA ROR is upregulated in *in vitro* cultured hypertrophic cardiomyocytes, which deteriorates myocardial hypertrophy into cardiac hypertrophy and even HF [10]. Further, the ROR/miR-124-3p/TRAF6 axis regulated the ischemia reperfusion injury-induced inflammatory response in human cardiomyocytes [11]. Besides, overexpressed ROR promotes the biological characteristics of ox-LDL-induced HUVECs let-7b-5p/HOXA1 axis in atherosclerosis [12]. However, the importance of ROR in HF patients was unknown.

MicroRNAs (miRNAs) are endogenous, single-strand RNAs containing 22 nucleotides. Through complementary base pairing, miRNAs posttranscriptionally regulate target gene expressions [13]. miRNAs are extensively involved in cardiac pathophysiological process, including cardiac development, cardiac hypertrophy, myocardial ischemia, and HF [14–16]. The miR-125 family is highly conserved in mammals and participates in embryogenesis, immune response, tumorigenesis, and ischemia reperfusion injury [17, 18].

miR-125b is transcribed on chromosome 11q23 (has-miR-125b-1) and 21q21 (has-miR-125b-2) [19]. Busk and Cirera [20] suggested that miR-125b is downregulated in HF patients. Further, miR-125b is critical for fibroblast-to-myofibroblast transition and cardiac fibrosis [21]. In addition, hypoxia-elicited mesenchymal stem cell-derived exosomes facilitate cardiac repair through miR-125b-mediated prevention of cell death in myocardial infarction [22]. However, the role of miR-125b in heart failure was unclear. In this paper, we aim to uncover the prognostic potentials of lncRNA ROR and miR-125b in HF patients combined ARF.

## 2. Patients and Methods

### 2.1. Baseline Characteristics

A total of 90 HF patients combined ARF treated in our hospital from April 2016 to December 2018 were included. Based on the New York Heart Association (NYHA) functional classification, there were 0 case in class I, 30 in class II, 32 in class III, and 28 in class IV. NYHA is classified into four categories according to limited levels of physical activities. Class I: physical activity is not limited. Class II: physical activity in patients with heart diseases is slightly limited with fatigue, palpitation, and dyspnea. Class III: physical activity is markedly limited and comfortable at rest. Class IV: unable to carry out normal physical activity.

A total of 90 healthy subjects undergoing physical examination in our hospital during the same period were included as controls. Subjects with (1) no urine; (2) endocrine diseases, skeletal muscle diseases, immune diseases, and malignancies; and (3) mental disorders were excluded. This study was approved by the Ethics Committee of the First Affiliated Hospital of Hebei North University. Signed written informed consents were obtained from all participants before the study.

### 2.2. Sample Collection

5 mL of venous blood was extracted in each subject under the fasting state in the morning. Blood was centrifuged at 3000 r/min for 10 min, and the serum was collected and stored at -80°C.

### 2.3. Quantitative Real-Time Polymerase Chain Reaction (qRT-PCR)

TRIzol method (Invitrogen, Carlsbad, CA, USA) was applied for isolating RNAs from serum samples. Through reverse transcription of RNA, the extracted complementary deoxyribonucleic acid (cDNA) was used for PCR detection by SYBR Green method (TaKaRa, Tokyo, Japan). Primer sequences were listed as follows: lncRNA ROR, F: 5′-CGAACGAGAGGACCGAAG-3′, R: 5′-GCCAAGTTCTAGATAAGC-3′; GAPDH, F: 5′-ACGGCAAGTTCAACGGCACAG-3′, R: 5′-GACGCCAGTAGACTCCACGACA-3′; miR-125b, F: 5′-GATCTGCAGCTCTCCCAGGGGCTGGCTTCAG-3′, R: 5′-GATCATATGGAGGCAGAAAGGATGGAG-3′; U6, F: 5′-CTCGCTTCGGCAGCACATATACT-3′, R: 5′-ACGCTTCACGAATTTGCGTGTC-3′.

### 2.4. Follow-Up

All patients were followed up through telephone, outpatient review, hospitalized investigation, or other methods for 24 months with 6 months interval. Disease onset, rehospitalization, and death were recorded.

### 2.5. Statistical Analysis

Statistical Product and Service Solutions (SPSS) 20.0 (IBM, Armonk, NY, USA) was used for all statistical analysis. Data were expressed as mean ± SD (standard deviation). Differences between two groups were analyzed by using the Student *t*-test. Comparison between multiple groups was done using one-way ANOVA test followed by post hoc test (least significant difference). Pearson correlation test was applied for assessing the relationship between serum levels of lncRNA ROR and miR-125b. Diagnostic potentials were assessed by depicting receiver operating characteristic (ROC) curves. *p* < 0.05 indicated the significant difference.

## 3. Results

### 3.1. Baseline Characteristics of Subjects

Through analyzing clinical data of subjects, no significant differences were found in age, sex, and BMI between healthy subjects and HF patients combined ARF (Table 1). Baseline characteristics of them were comparable.

### 3.2. Serum Levels of lncRNA ROR and miR-125b

Compared with healthy subjects, serum level of lncRNA ROR was upregulated in HF patients combined ARF (Figure 1(a)), while miR-125b level was downregulated (Figure 1(b)).

### 3.3. Correlation between Serum Levels of lncRNA ROR and miR-125b with NYHA

There were 0 case in NYHA class I, 30 in class II, 32 in class III, and 28 in class IV included in this trial. Interestingly, serum level of lncRNA ROR gradually increased with NYHA worsening in HF patients combined ARF (Figure 2(a)). Conversely, miR-125b level showed the opposite trend (Figure 2(b)). It is believed that high level of lncRNA ROR and low level of miR-125b aggravated the development of HF.

### 3.4. Correlation between Serum Levels of lncRNA ROR and miR-125b

Pearson correlation test uncovered a negative link between serum levels of lncRNA ROR and miR-125b in HF patients combined ARF (Figure 3).

### 3.5. Diagnostic Potentials of lncRNA ROR and miR-125b in HF Combined ARF

ROC curves were depicted for assessing the potentials of lncRNA ROR and miR-125b as diagnostic biomarkers in HF combined ARF. As the data revealed, lncRNA ROR and miR-125b were qualified in diagnosing HF combined ARF (lncRNA ROR: AUC = 0.9199, cutoff value = 5.595, sensitivity = 92.22%, and specificity = 73.33%; miR-125b: AUC = 0.8509, cutoff value = 2.290, sensitivity = 81.11%, and specificity = 74.44%) (Figures 4(a) and 4(b)).

### 3.6. Correlation between Serum Levels of lncRNA ROR and miR-125b with Prognosis in HF Combined ARF

Based on the mentioned cutoff value of lncRNA ROR, included patients were assigned into two groups. After 2-year follow-up, 16 cases were dead. Higher incidences of death and rehospitalization were observed in HF combined ARF cases expressing higher serum level of lncRNA ROR. In a similar way, patients were assigned into two groups according to the cutoff value of miR-125b. HF patients combined ARF expressing lower level of miR-125b had higher incidences of death and rehospitalization (Table 2).

## 4. Discussion

Renal insufficiency secondary to HF is commonly seen and its mortality is high [23]. ARF is a key factor in determining the progression and prognosis of HF [24]. Recently, biomarkers of impaired renal function have been identified as risk factors for HF, displaying a predictive value for poor, long-term prognosis [25].

Critical functions of lncRNAs have been highlighted [26, 27]. Yang et al. [28] discovered differentially expressed lncRNAs between ischemic HF patients and nonischemic HF ones by RNA-seq. It is reported that lncRNA Mhrt 779 antagonizes the development of cardiac hypertrophy and HF in mice induced by aortic contraction [29]. miRNAs are highly conserved in different species and tissue-specific. Primary transcripts are cleaved into pre-miRNAs and then translocate into nuclei to form mature miRNAs [30, 31]. About 30% of human genomes can be regulated by miRNAs [9]. Scrutinio et al. [32] found downregulated miR⁃150⁃5p in advanced HF patients, which is linked to cardiac remodeling, disease severity, and prognosis. To uncover the role of ROR and miR-125b, compared to previous research, we found that lncRNA ROR was upregulated in serum of HF patients combined ARF; however, miR-125b was found to be downregulated in serum of HF combined ARF. Further, ROR increased as disease stage advanced while miR-125b showed an opposite phenotype. The previous findings indicated the potential relation between ROR and miR-125b in HF combined ARF. lncRNA-miRNA interaction contributes to cell phenotype regulations [33]. Through absorbing miRNAs as ceRNAs, lncRNAs inhibit miRNA expressions [34]. Besides, lncRNAs are precursors of miRNAs through intracellular cleavage [35]. GAS5 is downregulated in fibrotic cardiac tissues, which alleviates HF by negatively regulating miR-21 [36]. Upregulated HOTAIR may be a biomarker of HF [37]. HOTAIR regulates phosphatase and tensin homologue expressions in HF by competing with miR-19 [38]. Through Pearson correlation test, we found that lncRNA ROR was negatively linked to miR-125b in serum of HF patients combined ARF.

Circulating lncRNA could act as a prognostic factor for disease. In previous study, NEAT1 was reported as an unfavorable prognostic factor in chronic heart failure patients by log-rank test and ROC analysis [39]. Further, Chen et al. also found that NEAT1 was an unfavorable factor in acute ST-segment elevation myocardial infarction by ROC analysis [40]. In our research, we found that ROR and miR-125b were prognostic factors by ROC analysis.

However, there are still limitations in our research. This research only detected the level of ROR and miR-125b in clinical samples; thus, the in vivo and in vitro assays should be conducted to further explore the relationship of ROR and mirR-125b and HF. Moreover, their diagnostic and prognostic potentials in HF combined ARF were identified as well.

## 5. Conclusions

Serum level of lncRNA ROR is upregulated, and miR-125b is downregulated in HF patients combined ARF. Their levels are linked to NYHA classification, which can be utilized as prognostic biomarkers in HF combined ARF.

## Figures and Tables

**Figure 1:** Serum levels of lncRNA ROR and miR-125b. Serum levels of (a) lncRNA ROR and (b) miR-125b in healthy subjects and heart failure patients combined acute renal failure.

**Figure 2:** Correlation between serum levels of lncRNA ROR and miR-125b with NYHA. Serum levels of (a) lncRNA ROR and (b) miR-125b in heart failure patients combined acute renal failure with NYHA classes II, III, and IV.

**Figure 3:** Correlation between serum levels of lncRNA ROR and miR-125b. A negative link between serum levels of lncRNA ROR and miR-125b in heart failure patients combined acute renal failure.

**Figure 4:** Diagnostic potentials of lncRNA ROR and miR-125b in heart failure combined ARF. (a) Diagnostic potential of lncRNA ROR in heart failure patients combined acute renal failure (AUC = 0.9199, cutoff value = 5.595, sensitivity = 92.22%, and specificity = 73.33%). (b) Diagnostic potential of miR-125b in heart failure patients combined acute renal failure (AUC = 0.8509, cutoff value = 2.290, sensitivity = 81.11%, and specificity = 74.44%).

**Table 1:** Baseline characteristics of subjects.

Variable	Control	HF combined ARF	*p*
Age	62.13 ± 6.75	60.93 ± 5.85	0.204
Sex (male/female)	45/45	45/45	N.S.
BMI (kg/m^2^)	22.62 ± 3.11	22.73 ± 3.51	0.824

HF: heart failure; ARF: acute renal failure; BMI: body mass index; N.S.: no significant difference.

**Table 2:** Correlation between serum levels of lncRNA ROR and miR-125b with prognosis in heart failure combined ARF.

Variable	Death	Rehospitalization	Nonhospitalized
lncRNA ROR			
Low level (*n* = 36)	4	12	20
High level (*n* = 54)	12	33	9
*χ* ^2^		55.573	
*p*		<0.001	
miR-125b			
Low level (*n* = 58)	13	34	11
High level (*n* = 32)	3	11	18
*χ* ^2^		52.874	
*p*		<0.001	

## Data Availability

The datasets used and analyzed during the current study are available from the corresponding author on reasonable request.
